# Effectiveness and Safety of Low Dose of Tenofovir Disoproxil Fumarate in Malagasy Patients with Chronic Hepatitis B

**DOI:** 10.1155/2022/1654620

**Published:** 2022-05-31

**Authors:** Chantelli Iamblaudiot Razafindrazoto, Tovo Harimanana Rabenjanahary, Andry Lalaina Rinà Rakotozafindrabe, Sedera Radoniaina Rakotondrasoa, Nitah Harivony Randriamifidy, Anjaramalala Sitraka Rasolonjatovo, Soloniaina Hélio Razafimahefa, Rado Manitrala Ramanampamonjy

**Affiliations:** ^1^Department of Gastroenterology, University Hospital Joseph Raseta Befelatanana, Antananarivo, Madagascar; ^2^Faculty of Medicine, University of Antananarivo, Madagascar; ^3^Department of Hepato-Gastroenterology, University Hospital Andrainjato, Fianarantsoa, Madagascar; ^4^Faculty of Medicine, University of Fianarantsoa, Madagascar

## Abstract

**Background:**

Accessibility of full dose daily of tenofovir disoproxil fumarate (TDF) is limited in Madagascar with an estimated cost well above the purchasing power of Malagasy population.

**Objective:**

The study is aimed at evaluating the efficacy and safety of low-dose tenofovir for the treatment of chronic hepatitis B (CHB).

**Methods:**

This prospective cohort study from January 2018 to December 2020 was conducted in the Department of Hepato-Gastroenterology, University Hospital Joseph Raseta Befelatanana, Antananarivo, Madagascar. The patients enrolled in the study received low dose of TDF 900 mg/week (300 mg daily, three days per week).

**Results:**

A total of 45 patients (male/female: 31/14) were included. The mean age was 45.1 ± 11.5 years. Fifteen patients were nucleos(t)ide (NA)-naïve, and 30 patients had prior NA therapy (NA-experienced). Thirty patients were HBeAg positive. A complete virological response (CVR) was achieved in 36/45 patients (80%) at 3 months, 41/45 (91.1%) at 6 months, and 43/45 (95.6%) at 12 months. High viral load at baseline was negative predictive factor of CVR at 3 months (HR: 0.14; 95% CI: 0.022–0.92; *p*: 0.041). There was no significant difference in response between HBeAg-positive and HBeAg-negative patients, NA-naïve and NA-experienced patients, and cirrhotic and noncirrhotic patients. Low dose of tenofovir was well tolerated. Ten patients (22.22%) had mild side effects. Mild renal failure was observed in 3 patients (6.7%) during follow-up.

**Conclusion:**

Low dose of tenofovir is effective, safe, and well tolerated in a Malagasy population sample. These results still require verification in a large population.

## 1. Background

Hepatitis B virus (HBV) infection is a serious public health problem worldwide. Word Health Organization (WHO) estimates that 296 million people were living with chronic hepatitis B infection in 2019, with 1.5 million new infections each year. In 2019, hepatitis B resulted in an estimated 820,000 deaths, mostly from cirrhosis and hepatocellular carcinoma (HCC) [1, 2]. Madagascar is at a high-intermediate level of endemicity of HBV infection, according to the WHO classification, with a weighted prevalence of 6.9% [3]. Nucleoside/nucleotide analogs (NAs), which inhibit reverse transcription by HBV polymerase, are an important class of drugs that changed the treatment paradigm and prognosis of chronic hepatitis B (CHB) [4]. Lamivudine, the first oral antiviral agent approved to treat HBV, has a high risk development of resistant HBV mutants and viral breakthrough. Resistance to lamivudine emerges in approximately 75% of patients after 5 years of treatment (annual incidence: 15%) [5]. Tenofovir disoproxil fumarate (TDF) is a potent nucleotide analog recommended as first-line therapy for HVB-infected patients in recently published guidelines [4]. TDF has been shown effective in patients with resistance of lamivudine. No drug resistance to TDF has been observed [5]. However, the use of TDF, either as alternative to lamivudine or as a first-line treatment for CHB, is limited in Madagascar with an estimated cost well above the purchasing power of Malagasy population. According the new studies, a low dose of TDF preserved renal function and maintain viral suppression in patients with CHB, even those with advanced liver disease [6, 7]. The study is aimed at evaluating the efficacy and safety of low dose of TDF in the treatment of CHB.

## 2. Patients and Methods

### 2.1. Study Design, Period, and Settings

This was a prospective cohort study conducted in Gastroenterology Unit, University Hospital Joseph Raseta Befelatanana, Antananarivo, Madagascar, from January 2018 to December 2020.

### 2.2. Study Population

Patients with CHB (positive for serum HBV surface antigen for at least 6 months), treatment-naïve or treatment-experienced, hepatitis B e Antigen (HBeAg) negative, or HBeAg-positive, seen in outpatient, were consecutively enrolled. The patients enrolled in the study received low dose of TDF 900 mg/week (300 mg daily, three days per week).

The inclusion criteria were as follows: (1) patient males and nonpregnant and nonlactation females aged ≥18 years; (2) viral load ≥ 2000 IU/mL for HBeAg-negative and ≥20,000 IU/mL for HBeAg-positive in treatment-naïve patients; (3) previous treatment by lamivudine or full-dose TDF for more than 3 months, viraemic or nonviraemic in NA-experienced patients; and (4) patients with cirrhosis or fibrosis F3/F4.

The exclusion criteria were as follows: (1) eGFR < 50 ml/min/1.73 m^2^; (2) evidence of HCC or other malignancy; (3) coinfection with human immunodeficiency virus, hepatitis C virus, and hepatitis D virus; (4) presence of severe comorbidities; (5) follow − up duration < 12 months; and (6) absence viral load monitoring during follow-up.

### 2.3. Methods

Demographic and laboratory data including age, sex, anti-HBV treatment history, fibrosis status, serum HBV-DNA levels, and HBeAg; serum alanine aminotransferase (ALT); serum creatinine, estimated glomerular filtration rate (eGFR) calculated by Chronic Kidney Disease Epidemiology Collaboration equation; and adverse events (AEs) were collected. The data were divided into 3 categories: treatment-naïve, experienced viraemic, and experienced nonviraemic patients.

A diagnosis of cirrhosis was based on the results of noninvasive liver examination (clinical, hepatobiliary ultrasound, and degree of fibrosis). Fibrosis was evaluated using FibroTest®, which applies four stages of increasing severity (F0 corresponds to an absence of fibrosis, while F4 corresponds to cirrhosis). The HBV-DNA levels were ascertained by real-time PCR (Cobas 8800 Roche Real-Time PCR, Cerba, France), with a lower limit of quantification of 20 IU/mL.

The patients enrolled in the study received low dose of TDF, 300 mg daily, three days per week (900 mg/week). All of the patients were followed up periodically (every 3 or 6 months). Viral load, ALT, serum creatinine level, and serum phosphorus level were measured before the initiation of treatment and then monitored every 3 months to evaluate efficacy and safety of low dose of TDF. For HCC screening, all patients underwent abdominal ultrasound and alpha-fetoprotein every 6 months. All adverse events reported by the patient or observed during the treatment period were recorded during follow-up. In case of severe renal failure (eGFR < 30 ml/min/1.73 m^2^), (1) TDF was be switched to lamivudine for treatment-naïve patients and (2) temporary discontinuation of TDF with monitoring of viral load and serum creatinine levels every 3 months for prior NA-therapy patients.

### 2.4. Endpoints and Outcomes

The primary endpoint was complete virological response (CVR), defined as an HBV viral load of 20 IU/ml during treatment (3 months and/or 6 months and/or 12 months).

The secondary endpoints were biochemical response (ALT normalization during follow-up), partial virological response (HBV-DNA between 20 and 2000 IU/mL during treatment), and clinical responses (absence of HCC development and absence of decompensation in cirrhotics).

Tolerance was judged according to the presence of adverse events and nephrotoxicity during follow-up. The renal toxicity was defined as a decline in eGFR of ≥25% from baseline during treatment.

### 2.5. Statistical Analysis

Data were statistically analyzed using the SPSS version 25 software. Categorical variables were defined as proportion (%) and compared by Chi-square or Fisher's exact test. Continuous variables are mean ± standard deviation (SD) and were assessed by Student's *t*-test or Mann-Whitney-Wilcoxon *U* test. The multivariate analyses using Cox's proportional hazard and logistic regression model were adopted to determine the predictive factors for CVR. *p* value < 0.05 was considered statistically significant.

## 3. Results

### 3.1. Characteristics of the Study Populations

Of the 45 patients included, 31 (68.9%) were male with sex ratio of 2.2. The mean age was 45.1 ± 11.5 years (range: 21-70 years). HBV was discovered during routine screening in 75.6%. Seven patients (15.6%) were in the cirrhosis stage, including 4/7 (57.1%) Child-Pugh A patients and 3/7 (42.9%) Child-Pugh B patients. Fifteen patients (33.3%) were NA-naïve and 30 (66.7%) NA-experienced. In NA-experienced patients, 20 patients (44.4%) had been previously treated with lamivudine and 10 patients' (22.2%) full-dose of TDF. The majority of patients had a fibrosis F1 and F2 with a respective rate of 28.9% (*n* = 13) and 46.7% (*n* = 21). Thirty patients (66.7%) were HBeAg positive and 15 (33.3%) HBeAg negative. Mean plasma HBV DNA was 3.70 ± 1.81 log 10 IU/mL. The 10 patients previously treated with full dose of TDF had an undetectable viral load at baseline, and the remaining 35 patients (77.8%) were viraemic. Sixteen patients (35.6%) had elevated ALT levels at baseline. The mean ALT level was 54.8 ± 55.2 IU/L. The mean eGFR was 120.4 ± 20.2 ml/min/1.73 m^2^. The baseline characteristics of patients are shown in Table 1.

### 3.2. Virological, Biochemical, and Clinical Responses

Overall, a CVR was observed in 36/45 patients (80%) at 3 months, 41/45 (91.1%) at 6 months, and 43/45 (95.6%) at 12 months. In patients with viraemic at baseline, CVR was 74.3% (26/35) at 3 months, 88.6% (31/35) at 6 months, and 94.3% (33/35) at 12 months. All 10 nonviraemic patients at baseline (previously treated with full dose of TDF) had persistent undetectable HBV-DNA (<20 IU/mL) at 3, 6, and 12 months after low dose of TDF. ALT normalization was observed in 29/45 patients (64.4%) at 3 months, 39/45 (86.7%) at 6 months, and 45/45 (100%) at 12 months. In patients with elevated ALT at baseline, ALT normalization was observed in 0% (0/16) at 3 months, 62.5% (10/16) at 6 months, and 100% (16/16) at 12 months. No HCC development and no cirrhotic decompensation were observed during follow-up. Virological, biochemical and clinical responses are shown in Tables 2 and 3. There was no significant difference in response (CVR and ALT normalization) between HBeAg-positive and HBeAg-negative, NA-naïve and NA-experienced, and cirrhotic and noncirrhotic patients at 3, 6, and 12 months. High viral load (HBV − DNA ≥ 20,000 IU/mL) at baseline was negative predictive factor of CVR at 3 months by Cox regression analysis (HR: 0.14; CI: 0.022-0.92; *p*: 0.041) (Table 4).

### 3.3. Tolerance and Adverse Events

Thirty-five patients (77.8%) had good tolerance to low dose of TDF. Ten patients (22.2%) had mild side-effects. Asthenia, nausea, and abdominal pain were the most common side effects. Three patients (6.7%) had a renal toxicity with mild renal failure (eGFR > 50 mL/mn/1.73 m^2^), which remained stable during follow-up. All three patients were previously treated with full dose of TDF. The tolerance and side effects of patients are shown in Table 5.

## 4. Discussion

To our knowledge, this was the first study to evaluate the efficacy and safety of low dose of TDF in the Malagasy population. Nevertheless, this study is significant because there are few studies evaluating the virological response and tolerance of low dose of TDF in NA-naïve and NA-experienced CHB patients. This study will allow a considerable reduction in the cost of treatment and consequently will ensure good compliance in CHB patients in low-income countries such as Madagascar.

The CVR in this study ranged from 80 to 95.6% over a 3 to 12-month treatment period. In addition, in all NA-experienced nonviraemic patients, the viral load was maintained undetectable during low-dose TDF treatment. There was no significant difference in response between HBeAg-positive and HBeAg-negative, NA-naïve and NA-experienced, and cirrhotic and noncirrhotic patients. These results confirm the efficacy of low-dose TDF in controlling HBV viremia and also the high barrier to resistance of this drug, even at low dose. According to the new studies, low-dose TDF could help maintain viral suppression in patients with chronic hepatitis B virus infection, even those with advanced liver disease [6, 7]. An Italian open-label clinical trial showed persistent viral suppression in 10 of 11 patients who received low-dose TDF (75 mg daily) for a prolonged period without emergence of resistance and remains more potent than adefovir at the standard dose [6]. A US study of 69 patients showed persistence of viral suppression in all patients on low-dose TDF (75-300 mg Q48h) [7]. These authors suggested this protocol for low-income countries as it could reduce the cost of therapy [6, 7]. However, according to the data from this study, CVR was achieved rapidly in patients with a viral load < 20,000 IU/mL, whereas it takes longer to achieve undetectable viral load in patients with a viral load > 20,000 IU/mL. We also found that CVR was higher in experienced than naïve patients. Therefore, we suggest that this protocol remains an alternative in patients on lamivudine with viral load rebound and cannot benefit from full-dose tenofovir due to its high cost. Low-dose TDF can also be offered to patients treated with full-dose tenofovir and nonviraemic.

The rate of CVR at 48 weeks in patients receiving a low dose of TDF in our study was similar and consistent with data from the literature including patients on full-dose tenofovir. Sehonou et al. (Benin, 2018) observed a CVR of 92.6% at 48 weeks [8]. Pan et al. [9] in a 2015 US study of 512 patients including 217 Asians and 299 non-Asians had found 96% and 97%, respectively, in Asian and non-Asian patients as the rate of CVR after 48 weeks. Marcellin et al. [10] (2016 in Clichy, France) had reported 92% CVR at 12 months. Nevertheless, several studies had reported virological response rates far below ours after 48 weeks of treatment. Wang et al., in a meta-analysis of 5 studies containing 633 patients, reported a CVR of 81.5% after 48 weeks of treatment [11–16]. Yu et al. (South Korea, 2015) had found a CVR ranging from 44.9 to 89.6% over 3 to 12 months [17]. The mean viral load at inclusion of our patients was very low (3.7 log_10_) compared to other studies (>5 log_10_ on average) explaining our high CVR rate. In addition, the majority of NA-experienced patients with full-dose TDF were nonviraemic at the time of inclusion in the study. Therefore, a long-term study in NA-naïve patients with a very high viral load will be necessary. High viral load at baseline was a negative predictive of CVR (HR: 0.14; CI: 0.022-0.92; *p* = 0.041). This finding has been reported by the majority of studies [2, 17–19].

In the present study, no cases of HCC and cirrhotic decompensation occurred during follow-up. This is probably due to the relatively short duration of follow-up in our study. However, TDF treatment decreases the risk of HCC but does not completely negate it. Liu et al. [20], in 2019, had objectified that TDF was independently associated with reduced risk of HCC (aHR 0.46, *p* < 0.01), decompensation (aHR 0.28, *p* = 0.01), and death (aHR 0.06, *p* < 0.01).

A low dose of TDF was well tolerated in this Malagasy population sample, with no unexpected side effects. Asthenia, nausea, and abdominal pain were the most common side effects. In controlled clinical trials in patients with CHB, more patients treated with tenofovir experienced nausea (9% tenofovir versus 2% adefovir) [21]. Other common side effects including abdominal pain, diarrhea, headache, dizziness, fatigue, nasopharyngitis, back pain, and rash occurred in more than 5% [21]. The safety profile of TDF in this study was similar to that reported in clinical trials and in other field studies performed in a larger population [2, 7–22]. Our study reported the renal toxicity (mild renal failure) in 3/45 patients (6.7%) at 12 months of treatment. All three patients were previously treated with full-dose tenofovir. A significant decrease in eGFR was observed in our patients at 12 months of low dose of TDF (104.3 ± 25.2 vs 120.4 ± 20.2, *p* = 0.001). Lieng et al. [7] reported that the low dose of TDF preserved renal function. These authors also found an improvement in renal failure in patients pretreated with full-dose TDF during the first year of low dose of TDF, and this renal failure remained stable thereafter [7].

## 5. Limitation of the Study

The study had several limitations. The main limitations were the short duration of the study and the nonhomogeneity of population study which restricted the validity of our results to certain groups of patients.

## 6. Conclusion

This study is a first in Madagascar on the efficacy of a low dose of tenofovir. Despite the limitations of the study, low dose of tenofovir effectively maintains CVR in NA-naïve and NA-experienced patients with low viremia. A high level of HBV-DNA at baseline was a negative predictor of achieving CVR. A low dose of tenofovir is safe and well tolerated in treatment-naïve, pretreated, cirrhotic chronic HBV. Further research in a larger, long-term sample is needed to support our findings. A study evaluating low dose of tenofovir use in cirrhotic and/or high viral load patients seems essential based on our results.

## Figures and Tables

**Table 1:** Baseline characteristics of patients.

Characteristics	Total population (*n* = 45)	NA-naïve (*n* = 15)	NA-experienced, viraemic (*n* = 20)	NA-experienced, nonviraemic (*n* = 10)
Gender, male, *n* (%)	31 (68.9)	11 (73.3)	15 (75)	5 (50)
Age (years), means (SD)	45.1 (11.5)	41 (13)	46 (10)	48 (12)
Age range (years), *n* (%)				
<50	31 (68.9)	13 (86.7)	13 (65)	5 (50)
≥50	14 (31.1)	2 (13.3)	7 (35)	5 (50)
Hypertension, *n* (%)	5 (11,1)	3 (20)	1 (5)	1 (10)
Diabetes, *n* (%)	4 (8.9)	3 (20)	0 (0)	1 (10)
Methods of HBV discovery, *n* (%)				
Routine screening	34 (75.6)	10 (66.7)	18 (90)	6 (60)
Etiological work-up chronic liver disease	7 (15.6)	3 (20)	0 (0)	4 (40)
Disturbances in liver tests	4 (8.9)	2 (13.3)	2 (10)	0 (0)
HBeAg positive	30 (66.7)	10 (66.7)	17 (85)	3 (30)
HBeAg negative	15 (33.3)	5 (33.3)	3 (15)	7 (70)
Fibrosis status, *n* (%)				
F0	3 (6.7)	2 (13.3)	1 (5)	0 (0)
F1	13 (28.9)	5 (33.3)	6 (30)	2 (20)
F2	21 (46.7)	5 (33.3)	12 (60)	4 (40)
F3	1 (2.2)	0 (0)	1 (5)	0 (0)
F4	7 (15.6)	3 (20)	0 (0)	4 (40)
Cirrhosis, *n* (%)	7 (15.6)	3 (20)	0 (0)	4 (40)
Child-Pugh class (*n* = 7), *n* (%)				
A	4 (57.1)	2 (66.7)	0 (0)	2 (50)
B	3 (42.9)	1 (33.3)	0 (0)	2 (50)
C	0 (0)	0 (0)	0 (0)	0 (0)
HBV-DNA (IU/mL)				
<2000	13 (28.9)	0 (0)	3 (15)	10 (100)
2000–20,000	17 (37.8)	7 (46.7)	10 (50)	0 (0)
>20,000	15 (33.3)	8 (53.3)	7 (35)	0 (0)
High viral load (>1,000,000 IU/mL), *n* (%)	5 (11.1)	3 (20)	2 (10)	0 (0)
Undetectable viral load (<20 IU/mL), *n* (%)	10 (22.2)	0 (0)	0 (0)	10 (100)
Means HBV-DNA (SD) (log_10_ IU/mL)	3.7 (1.8)	4.8 (1.2)	4.2 (1.2)	1 (0)
ALT (IU/L), means (SD)	54.8 (55.2)	76 (83)	52 (35)	27 (7)
<40	29 (64.4)	9 (60)	10 (50)	10 (100)
40–80	8 (17.8)	2 (13.3)	6 (30)	0 (0)
>80	8 (17.8)	4 (26.7)	4 (20)	0 (0)
Platelets (10^3^/mm^3^), means (SD)	241.6 (80.7)	255.9 (90.7)	266.2 (50.5)	170.9 (80.1)
INR, means (SD)	1.1 (0.1)	1.1 (0.1)	1 (0.1)	1.2 (0.2)
Serum creatinine level (*μ*mol/L), means (SD)	69 (14.3)	65 (14)	69 (13)	74 (17)
eGFR (ml/mn/1.73 m^2^), means (SD)	120.4 (20.2)	120 (15)	119 (21)	110 (22)
<60	0 (0)	0 (0)	0 (0)	0 (0)
60–89	7 (15.6)	0 (0)	4 (20)	3 (30)
>89	38 (84.4)	15 (100)	16 (80)	7 (70)
Treatment-naïve (NA-naïve), *n* (%)	15 (33.3)	15 (100)	-	-
Prior NA therapy (NA-experienced), *n* (%)				
Lamivudine	20 (44.4)	-	20 (100)	0 (0)
Full-dose tenofovir	10 (22.2)	-	0 (0)	10 (100)

HBeAg: hepatitis B e antigen; DNA: deoxyribonucleic acid; HBV: hepatitis B virus; ALT: alanine aminotransferase; INR: international normalized ratio; eGFR: estimated glomerular filtration rate; SD: standard deviation; NA: nucleos(t)ide analog.

**Table 2:** Virological, biochemical, and clinical response after low-dose TDF in overall population, viraemic, and nonviraemic patients at baseline.

Variables	3 months, *n* (%)	6 months, *n* (%)	12 months, *n* (%)
*Overall response (N* = 45)			
CVR	36 (80)	41 (91.1)	43 (95.6)
PVR (ADN-VHB 20–2000 UI/mL)	5 (11.1)	3 (6.7)	2 (4.4)
Viral load ≥ 2000 UI/mL	4 (8.9)	1 (2.2)	0 (0)
ALT normalization	29 (64.4)	39 (86.7)	45 (100)
HCC development	0 (0)	0 (0)	0 (0)
Decompensation of cirrhosis (*N* = 7)	0 (0)	0 (0)	0 (0)
*Viraemic patients at baseline* (*N* = 35)			
CVR	26/35 (74.3)	31/35 (88.6)	33/35 (94.3)
PVR (ADN-VHB 20–2000 UI/mL)	5/35 (14.3)	3/35 (8.6)	2/35 (5.7)
Viral load ≥ 2000 UI/mL	4/35 (11.4)	1/35 (2.8)	0/35 (0)
*Nonviraemic patients at baseline* (*N* = 10)			
CVR	10/10 (100)	10/10 (100)	10/10 (100)
*Elevated ALT at baseline* (*N* = 16)			
ALT normalization	0/16 (0)	10/16 (62.5)	16/16 (100)

CVR: complete virological response; PVR: partial virological response; DNA: deoxyribonucleic acid; HBV: hepatitis B virus; ALT: alanine aminotransferase; HCC: hepatocellular carcinoma.

**Table 3:** Virological and biochemical response after low dose of TDF in naïve and experienced patients.

Variables	NA-naïve (*N* = 15)	NA-experienced, viraemic (*N* = 20)	NA-experienced, nonviraemic (*N* = 10)
3 months			
CVR, *n* (%)	11 (73.3)	15 (75)	10 (100)
ALT normalization, *n* (%)	11 (73.3)	12 (60)	6 (60)
6 months			
CVR, *n* (%)	12 (80)	19 (95)	10 (100)
ALT normalization, *n* (%)	12 (80)	17 (85)	10 (100)
12 months			
CVR, *n* (%)	14 (93.3)	19 (95)	10 (100)
ALT normalization, *n* (%)	15 (100)	20 (100)	10 (100)

CVR: complete virological response; ALT: alanine aminotransferase; NA: nucleos(t)ide analog.

**Table 4:** Analysis of the predictive factors for a CVR after 3 months of TDF.

Variables	HR	CI (95%)	*p* value
Age			
[30–40[	0.35	0.07–1.55	0.167
[40–50[	0.38	0.10–1.49	0.165
[50–60[	0.48	0.10–2.20	0.345
[60–70[	0.33	0.05–1.50	0.99
Gender, female	0.67	0.25–1.59	0.365
Fibrosis status			
F1	1.83	0.29–11.40	0.515
F2	2.00	0.32–12.65	0.462
F3	1.77	0.11–27.45	0.654
F4	1.83	0.22–15.60	0.679
HBV-DNA (IU/mL)			
2000–20,000	0.95	0.15–4.97	0.945
≥20,000	0.14	0.02–0.92	0.041
ALT (IU/L)			
[40-80[	0.93	0.30–2.57	0.599
≥80	0.76	0.24–2.44	0.649
HBeAg-positive	0.83	0.28–2.45	0.731
NA-experienced therapy			
Lamivudine-experienced	0.74	0.26–2.13	0.65
Full-dose tenofovir experienced	0.88	0.10–7.65	0.905

HR: hazard ratio; CI: confidence interval; ALT: alanine aminotransferase; HBeAg: hepatitis B e antigen; NA: nucleos(t)ide analog.

**Table 5:** Tolerance and side effects of low dose of TDF.

Variables	Number of patients (%)
Severe side effects	0 (0)
Mild side effects	10 (22.2)
Nausea	5 (11.1)
Vomiting	2 (4.4)
Asthenia	10 (22.2)
Nasopharyngitis	1 (2.2)
Abdominal pain	5 (11.1)
Headache	2 (4.4)
Hypophosphatemia	0 (0)
Mild renal failure	3 (6.7)

## Data Availability

Data supporting the conclusions of this study are available from the corresponding author on reasonable request.

## Abbreviations

aHR: Adjusted hazard ratio
ALT: Alanine aminotransferase
CHB: Chronic hepatitis B
CVR: Complete virological response
DNA: Deoxyribonucleic acid
eGFR: Estimated glomerular filtration rate
HBeAg: Hepatitis B e antigen
HCC: Hepatocellular carcinoma
HR: Hazard ratio
HBV: Hepatitis B virus
INR: International normalized ratio
NA: Nucleos(t)ide analog
PVR: Partial virological response
SD: Standard deviation
TDF: Tenofovir disoproxil fumarate
WHO: World Health Organization.
